The article "Evaluation of a robot-assisted video-assisted thoracoscopic surgery programme" was retracted in 2015. Reason: fabricated or falsified data.

# Evaluation of a robot-assisted video-assisted thoracoscopic surgery programme

**DOI:** 10.3892/etm.2014.1532

**Published:** 2014-02-10

**Authors:** YONG HE, AMANS COONAR, SABIN GELVEZ-ZAPATA, POST SASTRY, ARCHER PAGE

**Affiliations:** 1 Department of Thoracic Surgery, The Fifth Hospital of Dalian, Dalian, Liaoning 116021, P.R. China; 2 Department of Thoracic Surgery, Papworth Hospital NHS Foundation Trust, Cambridge University Partners, Cambridge CB23 3RE, UK

**Keywords:** robot-assisted video-assisted thoracoscopic surgery, FreeHand, thoracoscopic camera holders

## Abstract

At present, there is increasing interest in surgical procedures using a robot-assisted device. The aim of this study was to investigate whether robot-assisted video-assisted thoracoscopic surgery (VATS) was more effective than conventional VATS. A total of 64 VATS lobectomies in Papworth Hospital (Cambridge, UK) were included in the study. In 34 cases the lobectomies were performed using conventional VATS (CV group), while in the remaining 30 cases the lobectomies were performed using robot-assisted VATS (Robotic group). In the robot-assisted VATS, FreeHand^®^, a thoracoscopic camera controller produced by Freehand 2010 Ltd. (Eastleigh, UK), was used. The duration of the thoracoscopic surgery in the Robotic group was 145.50±10.43 min, whereas in the CV group the duration was 162.79±9.40 min. The surgery duration in the Robotic group was 10.62% shorter than that in the CV group (P<0.05). The rates of bleeding, pulmonary infection, arrhythmia and prolonged air leak (≥5 days) in the Robotic group were 0, 3.33, 26.67 and 13.33%, respectively, while the corresponding rates in the CV group were 2.94, 5.88, 20.59 and 17.65%, respectively. No significant differences were identified in the postoperative complication rates between the two groups (P≥0.05). There was no perioperative mortality in the study. Compared with conventional VATS, FreeHand-assisted VATS provides a similar rate of postoperative complications and a reduced surgery duration, and may be beneficial for the recovery of the patients following VATS.

## Introduction

Video-assisted thoracoscopic surgery (VATS) is a challenging technical procedure in which the surgeon is required to demonstrate a high level of thoracoscopic skill and the role of the camera-holding assistant is important for the successful completion of the surgery. Prolonged procedures may be exhausting for the surgical team and manual camera control may be a source of frustration as a result of an unsteady visual field (1). By contrast, robotic camera holders may provide surgeons with a more stable image and enable them to control the view and direction (2).

The article "Evaluation of a robot-assisted video-assisted thoracoscopic surgery programme" was retracted in 2015. Reason: fabricated or falsified data.

At present, there is increasing interest in surgical procedures using a robot-assisted device. The advantages of using such a device include a steady, tremor-free image, the elimination of small inaccurate movements and decreased energy expenditure by the assistant (1). A number of studies have evaluated the advantages of robotic camera devices compared with manually controlled cameras or different types of devices (1,3–5). The Papworth Hospital (Cambridge, UK) has been the first to successfully complete a study involving robot-assisted VATS using the FreeHand^®^ device (Freehand 2010 Ltd., Eastleigh, UK). The results of the comparison between the two techniques are described in the present study.

## Subjects and methods

### Patients

A total of 64 VATS lobectomies were performed in Papworth Hospital from June to November 2012. In 30 cases the lobectomies were performed using robot-assisted VATS (Robotic group), while in the remaining 34 cases the lobectomies were performed using conventional VATS (CV group). In the Robotic group, there were 18 males and 12 females, and the patients had a mean age of 67.60±5.83 years; in the CV group, there were 19 males and 15 females (mean age, 68.08±5.69 years). There was no significant difference in the incidence of preoperative concurrent diseases between the two groups (P≥0.05; Table I). This study was conducted in accordance with the Declaration of Helsinki and with approval from the Ethics Committee of the Fifth Hospital of Dalian (Dalian, China) and Papworth Hospital NHS Foundation Trust (Cambridge, UK). Written informed consent was obtained from all participants.

### Device description

The FreeHand device, produced by Freehand 2010 Ltd (registration no. 000996343-002), is a thoracoscopic camera controller that may be used as an assistant device for VATS. FreeHand is suitable for use in all types of thoracoscopic procedure. The device consists of the following components: Control box, arm, hands-free control unit, indicator unit and foot pedal, in addition to a sterile, single-use pack and a FreeHand storage cart (Fig. 1).

Using the FreeHand device, the surgeon was in direct control of the scope position without the requirement for voice control or manipulation by an assistant. The scope was controlled by the hands-free controller, worn on a headband or attached to a surgical cap, and an activation pedal. The surgeon selected the direction of tilt and pan using head movements, and then initiated the movement using the activation pedal.

A Storz XENON 300 cold light projector (Karl Storz GmbH & Co. KG, Tuttlingen, Germany) was adopted for the programme.

### Statistical analysis

Data are presented as the mean ± standard error of the mean (SE). Statistical comparisons were conducted using χ^2^ and t-tests. P<0.05 was considered to indicate a statistically significant difference. All calculations were performed using SPSS version 12.0 statistical software for Windows (SPSS Inc., Chicago, IL, USA).

The article "Evaluation of a robot-assisted video-assisted thoracoscopic surgery programme" was retracted in 2015. Reason: fabricated or falsified data.

## Results

The complication rates were similar in the two groups. The rates of bleeding, pulmonary infection, arrhythmia and prolonged air leak (≥5 days) were 0, 3.33, 26.67 and 13.33%, respectively, in the Robotic group, while the rates of the corresponding complications in the CV group were 2.94, 5.88, 20.59 and 17.65%, respectively. There was no perioperative mortality in the study, and no significant differences were identified between the two groups with regard to the rates of postoperative complications (P≥0.05; Table II and Fig. 2).

The duration of the thoracoscopic surgery in the Robotic group was 145.50±10.43 min, whereas in the CV group the duration was 162.79±9.40 min. The surgery duration in the Robotic group was 10.62% shorter than that in the CV group (P<0.05; Table III).

## Discussion

Manually controlling the camera in thoracoscopic surgeries is a challenging task for the assistant. The experience of the camera-holding assistant is important for the surgical team and the surgical procedure as a whole. However, the individual assigned the role of holding the camera is usually a medical student or resident at the beginning of their thoracoscopic training, who may be unfamiliar with the surgical procedure, may be required to stand in an uncomfortable position and may become distracted. This may result in an unclear or unsteady visual field, which increases the rate of surgical errors. Surgical errors leading to injuries result predominantly from misperception, rather than lack of knowledge or judgment (6). The robotic camera holder is an attempt to overcome these disadvantages. Proponents of robotic devices have emphasised the enhanced technical ease of surgical procedures using them, owing to the advantages of the elimination of tremor (7,8).

There are a number robotic camera devices that have been applied in medicine. The FreeHand device, which was evaluated during the VATS procedures in the present study, is one type of robotic camera controller. FreeHand is a novel robot assistant device, produced by Freehand 2010 Ltd., which replaces the role of the camera-holding assistant. FreeHand enables an operator to move a robotic arm holding the video-scope by movement commands, thereby resulting in a good, stable view that is able to be held for a long time. The surgeon carries a small, lightweight headset. The movement of the camera is controlled by simple head movements, and the camera is activated by pressing a footswitch. With this system, unlike with human assistants, occasional movements of the camera, which move the target out of frame, are eliminated (9). The Automated Endoscope System for Optimal Positioning (AESOP; Intuitive Surgical, Inc., Sunnyvale, CA, USA) is one of the most popular robotic camera holders used during laparoscopic radical prostatectomy (10,11). The AESOP system was first used in urological surgery. The AESOP system has been suggested to be a feasible and effective tool for laparoscopic surgery by an experienced surgeon (12). AESOP responded to surgical voice commands to maneuver the camera, with the remainder of the procedure being performed with VATS techniques. In addition, a successful thoracoscopic surgery for lung cancer using a voice-controlled robot has been described (13,14). The EndoAssist (Armstrong Healthcare, High Wycombe, UK) is similar to the FreeHand in that it is controlled by the surgeon’s head movements; however, the device is cumbersome and is similar in size to a standard C-arm (1).

The article "Evaluation of a robot-assisted video-assisted thoracoscopic surgery programme" was retracted in 2015. Reason: fabricated or falsified data.

Robotic camera holders have been evaluated in surgical and laparoscopic procedures. A study by Nebot *et al* (15) compared the EndoAssist and AESOP. The results showed that EndoAssist was significantly faster at accomplishing the procedure, since voice recognition errors occurred in the AESOP cases. Wagner *et al* (1) also compared these two robotic camera holders during laparoscopic radical prostatectomy. The robot setup time and operative steps were timed and compared between the two devices. It was concluded that the two robotic camera holders appeared to be equally efficient with respect to surgical performance. The advantages of the EndoAssist included its accurate response and ability to provide the desired surgical view; its disadvantages included its large profile, lack of a table-mounted design and the need for pedal activation. Robotic camera holders and human assistants have also been compared. Stolzenburg *et al* (3) compared the FreeHand robotic camera holder with human assistants during endoscopic extraperitoneal radical prostatectomy. In the study, the procedure was divided into several steps, each of which was compared. It was revealed that the time taken for each step and the total duration of the procedure were similar for the FreeHand and the human assistants; however, the FreeHand provided accurate and rapid camera movements without compromising the outcome of the procedure. In another study, Uchal *et al* (5) concluded that robotic and human camera holders had similar impacts on quality and procedure efficacy in a simulated laparoscopic procedure. Quality was measured according to accuracy errors, tissue damage, sliding knots and leaks, whereas procedure efficacy was measured according to the duration of the surgery, as well as non-target-directed and dangerous actions.

The article "Evaluation of a robot-assisted video-assisted thoracoscopic surgery programme" was retracted in 2015. Reason: fabricated or falsified data.

The present study compared a similar VATS procedure using FreeHand and human camera-holding assistants. The majority of the previous studies on robot-assisted VATS have demonstrated that such robotic technology facilitates safer and more precise dissection of the lobes and/or sequestered tissue than conventional VATS, and is thus likely to result in a reduction in bleeding and fewer conversions to open surgery (16,17). However, in a randomised trial comparing robot-assisted and conventional VATS, morbidity rates, blood loss, surgery duration and hospital stay were similar for the two types of VATS, and there was no difference in the postoperative quality of life scores between the two groups (18). In addition, a number of small studies have failed to demonstrate the added value of robotics (19–22). In the present study, it was demonstrated that the surgery duration in the Robotic group was shorter than that in the manual group, which was not consistent with the previous studies. In the future, a comparison between the various robotic camera devices is required, in order to identify the most efficient device for use in medicine.

Lung lobectomy is a common procedure that presents a surgical challenge. At present, anatomical lung resections are predominantly performed with stapling devices by means of VATS (23). The Papworth Hospital in Cambridge (UK) has pioneered the use of FreeHand to perform VATS. Through the application of the device in the present study, the thoracoscopic surgery duration was significantly shortened compared with the surgery duration in the CV group. This indicated that the device avoided time-wasting as a result of its enhanced stability. Furthermore, the repeated removal of the device to clean the mirror was not necessary. With regard to complications, statistical analysis revealed no significant differences between the Robotic and CV groups. These results were consistent with those of previous studies (24–26).

Due to the fact that the anesthesia and the duration of the thoracic surgery have direct impacts on the postoperative recovery of patients, reducing the duration of VATS procedures is likely to be beneficial for patients. Thus, further studies into the application of FreeHand-assisted thoracoscopic surgery are required. These further assessments of the application value of this programme require a greater application and the analysis of samples.

With regard to the shortcomings of the present study, a larger number of cases and a more detailed comparison of the procedures would have provided more comparative data and improved the accuracy of the statistical analysis. As increasing numbers of surgeons gain experience with this method, the surgical technique is likely to become more stable, and the surgery duration is likely to be reduced, as indicated by the present results. The reduction in surgery duration obtained in the present study may be attributed to the close and stable view obtained by the VATS technique using the FreeHand system.

The article "Evaluation of a robot-assisted video-assisted thoracoscopic surgery programme" was retracted in 2015. Reason: fabricated or falsified data.

## Figures and Tables

**Figure 1:** The FreeHand device (Freehand 2010, Ltd., Eastleigh, UK), which is suitable for use in all thoracoscopic procedures. FreeHand consists of the following components: Control box, arm, hands-free control unit, indicator unit and foot pedal, as well as a sterile, single-use pack and a Freehand storage cart.

**Figure 2:** The rates of postoperative complications were similar in the two groups. In the Robotic group, the rates of bleeding, pulmonary infection, arrhythmia and prolonged air leak (≥5 days) were 0, 3.33, 26.67 and 13.33%, respectively. In the CV group, the rates of the corresponding complications were 2.94, 5.88, 20.59 and 17.65%, respectively. No significant differences were identified between the two groups (P≥0.05). Robotic group, robot-assisted video-assisted thoracoscopic surgery (VATS); CV group, conventional VATS.

**Table I:** Analysis of the preoperative concurrent diseases in the two groups.

Disease	Robotic group % (n)	CV group % (n)	χ^2^	P-value
Heart disease	36.67 (11/30)	38.24 (13/34)	0.017	0.897
Emphysema	26.67 (8/30)	20.59 (7/34)	0.328	0.567
Diabetes	20.00 (6/30)	20.59 (7/34)	0.003	0.953

Robotic group, robot-assisted video-assisted thoracoscopic surgery (VATS); CV group, conventional VATS.

**Table II:** Analysis of the postoperative complications in the two groups.

Complication	Robotic group % (n)	CV group % (n)	χ^2^	P-value
Bleeding	0 (0/30)	2.94 (1/34)	0.896	0.344
Pulmonary infection	3.33 (1/30)	5.88 (2/34)	0.232	0.630
Arrhythmia	26.67 (8/30)	20.59 (7/34)	0.328	0.567
Prolonged air leak	13.33 (4/30)	17.65 (6/34)	0.225	0.635

There was no perioperative mortality among the cases. Robotic group, robot-assisted video-assisted thoracoscopic surgery (VATS); CV group, conventional VATS.

**Table III:** Analysis of the average thoracoscopic surgery duration (min) in the two groups.

Robotic group	CV group	P-value
145.50±10.43	162.79±9.40	0.016

Robotic group, robot-assisted video-assisted thoracoscopic surgery (VATS); CV group, conventional VATS.
